# Hub Genes and Long Noncoding RNAs That Regulates It Associated with the Prognosis of Esophageal Squamous Cell Carcinoma Based on Bioinformatics Analysis

**DOI:** 10.1155/2022/6027058

**Published:** 2022-09-19

**Authors:** Jun Lu, Ruichao Li, Minghao Fang, Shun Ke

**Affiliations:** ^1^Department of Emergency Medicine & Intensive Care Unit, Tongji Hospital, Tongji Medical College, Huazhong University of Science and Technology, Wuhan 430030, China; ^2^Department of General Medicine, Tongji Hospital, Tongji Medical College, Huazhong University of Science and Technology, Wuhan 430030, China

## Abstract

**Objective:**

Through bioinformatics analysis methods, the public databases GEO and TCGA were used to research mRNA and squamous cell carcinoma of the esophagus, construct a lncRNA-mRNA network, and screen hub genes and lncRNAs related to prognosis.

**Method:**

Download esophageal squamous cell carcinoma-related mRNA and lncRNA datasets GEO and TCGA public datasets, as well as clinical data, use bioinformatic tools to perform gene differential expression analysis on the datasets to obtain differentially expressing mRNA (DEmRNA) and lncRNA (DElncRNA), and plot volcano plots and cluster heatmaps. The differential intersection of differentially expressed DEmRNA and DElncRNA was extracted by Venn diagram and imported into CytoScape software, a regulatory network visualization software, to construct a lncRNA-mRNA network and use cytoHubba and MCODE plug-ins to screen hub genes and key lncRNAs. The DEmRNA in the network was imported into the Gene and Protein Interaction Retrieval Database (STRING), gene-encoded protein–protein interactions (PPI) network maps were created, and the genes in the PPI network maps were submitted to GO functional annotation and pathway enrichment analysis using Kyoto Encyclopedia of Gene Genomes (KEGG) (KEGG). The link between hub gene and prognosis was studied using the clinical data collected by TCGA.

**Result:**

Retrieve the datasets GSE23400 and GSE38129 from the GEO database and the esophageal squamous cell carcinoma-related mRNAs from TCGA databases and then obtain intersection. Differentially regulated genes revealed a correlation of 326 (up) with 191 (down) in terms of the differential intersection; for this study, we need to collect the GSE130078 dataset from GEO, as well as the lncRNAs from TCGA databases that are connected to esophageal squamous cell cancer. There were 184 differentially up- and downregulated genes in the differential intersection. A differential intersection network of the differential intersection lncRNA-mRNA network allowed us to identify the hub genes, including COL5A2 (COL3A1), COL1A1 (COL1A1), CTD-2171N6.1 (CTD-2171N6.1), and RP11-863P13.3 (RP11-863P13.3). The extracellular matrix, which is important in protein digestion and absorption, was shown to be the primary site of functional enrichment, as shown by GO/KEGG analysis. Squamous cell carcinoma of the mouth and throat is associated with a poor prognosis because of a change in the extracellular matrix structure caused by specific long noncoding RNA (lncRNA) regulatory upregulation.

**Conclusion:**

For the purpose of predicting the prognosis of cancer of the esophagus, researchers studied the esophageal squamous cell carcinoma-related hub genes and important noncoding RNAs (ncRNAs).

## 1. Introduction

Eosophageal carcinoma (EC) is one of the most prevalent cancers in the world [1]. Cancer is the third most common and the fourth most deadly disease on China's mainland [2]. Esophageal squamous cell carcinoma (ESCC), which accounts for 90% of all esophageal cancer patients worldwide, is the most common pathological diagnosis [3]. Early ESCC patients had a five-year survival rate of up to 90%. According to the Centers for Disease Control and Prevention, 50 percent of ESCC patients in China have already had tumor metastases. Following surgical treatment, radiation therapy, and chemotherapy, survival rate after five years is under twenty percent [4, 5]. There is no doubt that the best chance of a cure lies on an early diagnosis and the presence of metastases in other parts of the body. Consequently, novel early screening markers and treatment targets are needed. It is thought that long noncoding RNA (lncRNA) plays an important role in tumor formation and growth because of its length of over 200 nucleotides [6]. Previous studies have shown that acute myeloid leukemia is characterized by a high degree of downregulation of the microRNA known as miR-192. It is able to influence tumor cell proliferation and cell cycle progression by interaction with cyclin CCNT2, which is responsible for regulating cell proliferation and cell cycle progression [7]. Esophageal squamous cell carcinoma has a decreased expression of long-chain noncoding NKILA that inhibits cell proliferation and migration by preventing the NF-B signaling pathway from activating [8]. The miR-7/HOXB13 axis can be activated by circular RNA CIRS-7 to increase the development and metabolism of esophageal squamous cell carcinoma [9]. Although noncoding RNAs (lncRNAs) have recently risen to the forefront of tumor formation and development studies, no studies have looked at lncRNAs as potential tumor indicators in esophageal squamous cell carcinoma.

As part of this study, we used the combined analysis of GEO and TCGA to screen out the differential expression profiles of long noncoding RNA (lncRNA) and short noncoding RNA (mRNA) in esophageal squamous cell carcinoma and constructed a network and selected hub genes using cytoscape. We then used clinical samples to verify the final prognosis of the hub gene and the feasibility as a prognostic marker for this type of cancer.

## 2. Materials and Methods

### 2.1. Data Collection

Esophageal squamous cell carcinoma-related mRNA and lncRNA datasets from the TCGA database can be downloaded from GSE23400, GSE38129, and GSE130078 gene probe matrices, respectively, from the Gene Expression Omnibus (GEO, http://www.ncbi.nlm.nih.gov/geo/), as well as GPL96, GPL571, and HiSeq 2000 annotation information file of the corresponding platform and then convert the probe IDs of the probe matrix in the dataset into the gene IDs and Ensembl gene IDs in the annotation information.

### 2.2. Differential Expression and Differential Intersection

Standard data were obtained by filtering and normalizing the data, and the log2 fold change (FC) absolute values of greater than 1.5 were used as a standard for differential gene screening. This allowed researchers to identify the mRNAs that were differentially expressed (DEmRNA) and lncRNAs that were differentially expressed (DElncRNA). DEmRNA and DElncRNA are the intersections of the datasets GSE23400 and GSE38129 and the mRNA- and lncRNA-related datasets in the TCGA database, respectively, taken from the intersection.

### 2.3. Construct lncRNA-mRNA Network and Protein-Protein Interaction Network Diagram

Introducing the intersection of DEmRNA and DElncRNA into cytoScape v3.7 [10] software, build lncRNA-mRNA network and use cytoHubba and MCODE plug-ins to obtain hub genes and key lncRNAs. Using the STRING [11] online tool, analyze the protein-protein interaction (PPI) through DEmRNA. Select Required Confidence (combined score) > 0.7 as the threshold for protein-protein interaction to construct a PPI network graph.

### 2.4. Enrichment Analysis and Survival Analysis

As a statistically significant function and signaling path, DEmRNA enrichment pathways are analyzed using GO functional annotation and Kyoto Encyclopedia of Genes and Genomes (KEGG) path analysis; a statistically significant result is one that has a *P* value that is less than 0.05. The survival curve between the hub gene and disease-free survival (DFS) was produced for prognostic analysis using esophageal squamous cell carcinoma survival data taken from the TCGA database. This was done in order to determine the likelihood of a favorable outcome.

### 2.5. Statistical Methods

Use R language limma or edgeR package [12] to calculate differential expression, and draw Venn diagram to take differential intersection. Through CytoScape software, build lncRNA-mRNA network to screen hub genes and key lncRNAs. Stitch together a PPI network with the help of the STRING database, and then, do a survival study using the Kaplan-Meier curve.

## 3. Results

### 3.1. DEmRNA and DElncRNA Screening Findings

DEmRNAs screened from the three datasets of GSE23400, GSE38129, and TCGA are shown in Table 1, and the number of DElncRNAs screened from the two datasets of GSE130078 and TCGA is shown in Table 2. Cluster analysis was performed on the screened differential genes marking the differential genes with significant differences, and cluster heatmaps and volcano maps were drawn (Figures 1(a) and 1(b)).

### 3.2. Difference Intersection and Venn Diagram

The intersection analysis of DEmRNA and DElncRNA indicated 326 differentially upregulated genes and 191 differentially downregulated genes, respectively. There were 184 differentially upregulated lncRNAs and 57 differentially downregulated lncRNAs. Then, a Venn diagram was constructed (Figures 2(a) and 2(b)).

### 3.3. Analysis of lncRNA-mRNA and PPI Network and Enrichment Results

A lncRNA-mRNA regulatory network was constructed with the help of CytoScape (Figure 3). Analyzing the established lncRNA-mRNA regulatory network indicated that lncRNA-RP11-863P13.3, RP11-576I22.2, and CTD-2171N6.1 can govern the upregulation of MMP11, THY1, and 16 more genes. MAMDC2-AS1 is the closest downregulated lncRNA related with gene regulation, interacting with 19 genes, including FHL1 and TGFBR3. Afterwards, using the online application STRING, a PPI network was constructed for the mRNAs that were the most directly influenced by lncRNAs. In addition, the hub genes were excluded from the analysis as a result of the connection degree of each gene (in this investigation, the top 10 genes with the highest connection degree were selected) (Figure 4(a)). It was shown that COL5A2, COL3A1, and COL1A1 as well as other hub genes had a greater influence on the lncRNA-mRNA regulatory network of esophageal squamous cell carcinoma than other hub genes. Biological process (BP), molecular function (MF), and cellular component (CC) are the three gene function categories identified by the GO and KEGG enrichment analyses of the genes in the aforementioned PPI network. The enrichment results revealed that the pathway with the highest enrichment score in BP was composed of extracellular matrix (Figure 4(b)), that the pathway with the highest enrichment score in CC was fibrillar collagen trimer (Figure 4(c)), and that the pathway with the highest enrichment score in MF is for the extracellular matrix structural components that confer tensile strength (Figure 4(d)). The protein digestion and absorption pathway received the greatest enrichment score according to KEGG (Figure 4(e)).

### 3.4. Survival Analysis

The selected hub genes of COL1A2, COL3A1, and COL5A2 were drawn using the Kaplan-Meier survival curve to analyze the clinical prognosis. These genes were chosen based on the clinical data provided by TCGA. It was discovered that all three of the hub genes, COL1A2, COL3A1, and COL5A2, had significant levels of expression. In addition, the disease-free survival duration of patients who had esophageal squamous cell carcinoma and had these hub genes in high expression was dramatically reduced (Figure 5). This suggests that it has certain clinical significance when determining the prognosis of patients who have esophageal squamous cell carcinoma.

## 4. Discussion

As we all know, little is known about the lncRNA signatures of HCC patients. One piece of study established six lncRNA signatures with the intention of predicting recurrence-free survival in HCC. Wu et al. then investigated these signatures in a specific HCC cohort in which the tumor may be removed [13, 14]. This research utilized lncRNA signatures to construct a lncRNA-mRNA interaction network in patients with esophageal squamous cell carcinoma. The researchers then screened interacting hub genes to predict survival, which is more accurate and clinically relevant than simply screening lncRNA features from the perspective of cellular function correlation. In this work, we examined the differential lncRNAs and mRNAs in esophageal squamous cell carcinoma and paracancerous tissue using a combined TCGA-GEO analysis and then calculated expression correlation between the above differential intersection lncRNA and differential intersection mRNA in TCGA data. After the lncRNA-mRNA relationship pair with the correlation coefficient greater than 0.7 was selected, we constructed the lncRNA-mRNA regulatory network with CytoScape. Subsequently, the STRING database was used to predict the hub gene to construct a PPI network to enrich the GO and KEGG pathways. We examined the influence of hub gene expression related with lncRNA on disease-free survival in esophageal squamous cell carcinoma using TCGA clinical prognostic data.

I is a fibrillar collagen found abundantly in bone, cornea, dermis, and tendon [15–17]. This gene is linked to osteogenesis imperfecta types I through IV, Ehlers-Danlos syndrome VIIA, classic Ehlers-Danlos syndrome, Caffey disease, and idiopathic osteoporosis. A reciprocal translocation between chromosomes 17 and 22, where this gene and the platelet-derived growth factor gene are situated, is related with dermatofibrosarcoma protuberans, a particular kind of skin tumor caused by aberrant production of growth factors. For this gene, two transcripts with alternate polyadenylation signals have been discovered [18–21]. In this study, clinical prognostic analysis based on TCGA revealed that the high expression of four genes, majority, caused by mutations, mount faucet, the faucet, and signs of abating, may considerably reduce the disease-free survival of esophageal squamous cell carcinoma and worsen the prognosis. These genes are COL1A1, COL1A2, COL3A1, and COL5A2. Therefore, we hypothesize that the high expression of the COL collagen family is associated with a worse prognosis for esophageal squamous cell carcinoma.

Extracellular matrix (ECM) is a type of insoluble structural component that mostly consists of collagen, elastin, proteoglycans, and glycoproteins. ECM can influence biological processes such as cell differentiation, proliferation, adhesion, morphogenesis, and phenotypic expression, according to studies [22]. Malignant tumor formation, progression, invasion, and metastasis are frequently accompanied by alterations in the extracellular matrix and expression of cell surface receptors [23]. Not only was the high level of LN and 61 significantly codistributed in human hepatocellular carcinoma (HCC) tissue but also the high level expression was negatively correlated with the prognosis of liver cancer patients, indicating that HCC cells may receive signals from LN via the 61 receptor, thereby causing the cancer to spread. Normal hepatocytes do not have a basement membrane and express the specific integrin family receptor 61 of laminin (LN). In the first stages of liver cancer's pathophysiology, portal vein invasion, intrahepatic metastasis, and extrahepatic metastases in the lungs and bones are common occurrences. The key aspects that decide a patient's prognosis with regard to liver cancer are the presence of invasion, metastasis, and postoperative recurrence of the disease. Matrix metalloproteinases, also known as MMPs, are responsible for the breakdown of extracellular matrix, also known as ECM. This is one of the most important links in the process of tumor cell invasion and metastasis. The presence of increased MMP levels and activity has been linked to a wide variety of cancerous tumors [24]. Among the GO annotation and KEGG pathway enrichment results, the related pathway of extracellular matrix property change has the highest enrichment score in extracellular matrix organization, fibrous collagen trimming, and extracellular matrix structure, indicating that COL collagen family represented by COL1A1 can result in a poor prognosis for patients by participating in the change of ECM properties to promote the generation and development of cancer cells. In this study, the pathway with the highest enrichment score in BP is extracellular matrix, the pathway with the highest enrichment score in CC is fibrillar collagen trimer, and the pathway with the highest enrichment score in MF is for the extracellular matrix structural components that confer tensile strength. The protein digestion and absorption pathway received the greatest enrichment score according to KEGG.

Epigenetics is a discipline of biology that investigates the heritable changes in gene expression and the stability of DNA sequence, which are necessary not only for the expansion and differentiation of cells but also for the occurrence and progression of cancers. DNA methylation, histone changes, and recently found noncoding RNAs are the key epigenetic processes [25]. Functional RNA molecules that cannot be translated into proteins are referred to as noncoding RNAs. Common regulatory noncoding RNAs include small interfering RNAs, microRNAs, piRNAs, and long noncoding RNAs [26]. Numerous studies have demonstrated that noncoding RNAs play an increasingly crucial role in epigenetic control. lncRNA participates in several biological processes, including the dose compensation effect, epigenetic control, cell cycle regulation, and cell differentiation regulation, among others, which play an important role, becoming a hot spot in genetics research. Tongji University used an integrated genomic data analysis method to research clinically relevant cancer lncRNAs and found two important prostate cancer lncRNA genes [27]. Studies have shown that lncRNA GLCC 1 binds to HSP 90 chaperones to form an RNA-protein complex, which stabilizes c-Myc in ubiquitination degradation in the cytoplasm to determine the transcription of its target gene LDHA and then to promote the genesis and glucose metabolism of colorectal cancer [28]. The interaction between HNF1A-AS1 and Egr1 promotes the ubiquitination and degradation of p21 that is mediated by CD34. This increases the expression of cyclin-dependent enzyme 2 (Kalindi kunj), kinases, and cyclin E1 and decreases the expression of p21, hence promoting the development of gastric cancer [6, 29]. These findings demonstrate that lncRNAs can influence gene expression via different pathways to mediate the evolution of tumor malignancy. This study revealed that the three noncoding RNA genes involved, engage in self, and CTD-2171N6.1 may upregulate the expression of the COL collagen family member COL1A1 and are also interconnected. Significant portions of the dataset are expressed in esophageal squamous cell carcinoma-affected tissues. Therefore, we examined whether lncRNA-RP11-863P13.3, RP11-576I22.2, and CTD-2171N6.1 may contribute to a poor prognosis in patients with esophageal squamous cell carcinoma by promoting the change of ECM characteristics through the upregulation of Exon 1, Ccl5, COL3A1, and fabricating. The lncRNA-mRNA regulatory network of esophageal squamous cell carcinoma had the most pronounced effect on the hub genes COL5A2, COL3A1, COL1A1, and others.

Bioinformatics analysis was used in this work to identify the COL collagen family genes and three critical lncRNAs associated with the poor clinical prognosis of esophageal squamous cell carcinoma. But we did not conduct in vitro and in vivo functional experiments to further analyze the mechanism due to all kinds of objective reasons, which is the biggest deficiency of this study. We will further study the expression regulation mechanism of related molecules in this study when the experimental conditions are met.

In conclusion, we have discovered three new lncRNAs as independent biological predictors of esophageal squamous cell carcinoma prognosis using bioinformatics, clinical data, and genetic profiles of thoroughly screened cohorts. To examine the progression process of ESCC and the particular mechanisms of action of these lncRNAs, however, it will be necessary to corroborate our findings in future research.

## Figures and Tables

**Figure 1:** (a) DEmRNA thermal map and volcano diagram. (b) Heatmap and volcano map of DElncRNA.

**Figure 2:** (a) Venn diagram of DEmRNA intersection. (b) Venn diagram of DElncRNA intersection.

**Figure 3:** Schematic of the lncRNA-mRNA regulation network.

**Figure 4:** Analysis of PPI network and hub gene enrichment.

**Figure 5:** Hub gene and DFS prognosis analysis.

**Table 1:** DEmRNA result statistics table.

Statistical information		Threshold dissimilarity		Gene variants		Samples	
Data sources	Platform	FC	*P*_value	Up	Down	Tumor	Normal
GSE23400	GPL96	1.5	0.05	614	570	53	53
GSE38129	GPL571	1.5	0.05	1056	990	30	30
TCGA	HTSeq	1.5	0.05	1417	1630	161	12

**Table 2:** DElncRNA.

Data information		Difference threshold		Differential number of lncRNAs		Number of samples	
Data sources	Platform	FC	*P*_value	Up	Down	Tumor	Normal
GSE130078	HiSeq 2000	1.5	0.05	512	302	Twenty-three	Twenty-three
TCGA	HTSeq	1.5	0.05	1266	1000	161	12

## Data Availability

The labeled dataset used to support the findings of this study is available from the corresponding author upon request.
